# The Diagnostic Value of Combined Detection of Serum Lp-PLA2 and Hcy and Color Doppler in Elderly Patients with Acute Coronary Syndrome and Effect on Endothelial Function

**DOI:** 10.1155/2022/3150670

**Published:** 2022-07-08

**Authors:** Li Zhao, Jingrui Qi, Fan Luo, Na Zhao

**Affiliations:** Cangzhou Central Hospital, Cangzhou, Hebei, China

## Abstract

**Objective:**

To evaluate the application value of serum lipoprotein-associated phospholipase A2 (Lp-PLA2) and homocysteine (Hcy) combined with color Doppler detection in elderly patients with acute coronary syndrome (ACS) and the influence on their endothelial function.

**Methods:**

From February 2019 to October 2020, 100 elderly patients with suspected ACS treated in our hospital were recruited and assigned (1 : 1) to a control group or an experimental group. The control group received color Doppler detection, and the experimental group received the combined detection of serum Lp-PLA2 and Hcy and color Doppler. Positive results were determined by the combined detection of the levels of LP-PLA2 and Hcy and color Doppler. The two groups were compared in terms of specificity, susceptibility, positive detection rate, negative detection rate, test accuracy, the area under the receiver operating characteristic (ROC) curve (AUC), the expression levels of interleukin-2 (IL-2), interleukin-12 (IL-12), interleukin-13 (IL-13), and the vascular endothelial function. The patients with ACS were divided into three subgroups according to the Gensini score three-quartile interval, and their Lp-PLA2 levels were calculated for analysis.

**Results:**

The test specificity, susceptibility, positive detection rate, negative detection rate, test accuracy, and AUC in the experimental group were much better than the those in the control group (all *P* < 0.05), and there were no significant differences in the expression levels of IL-2, IL-12, IL-13, and vascular endothelial function between the two groups (*P* > 0.05). The three subgroups showed similar levels of fasting blood glucose, total cholesterol, triglyceride, high-density lipoprotein-cholesterol, low-density lipoprotein-cholesterol, apolipoprotein A-I, glutamic-pyruvic transaminase, lutamic-oxaloacetic transaminase, homocysteine, and amino-terminal pro-brain natriuretic peptide (all *P* > 0.05). The severe condition group had the highest Lp-PLA2 level, followed by the moderate group, and then the mild group (*P* < 0.05). Moreover, the levels of LP-PLA2, aspartate transaminase (AST), and N-terminal pro hormone B-type natriuretic peptide (NT-proBNP) were all influencing factors for the coronary Gensini score (all *P* < 0.05).

**Conclusion:**

The combined detection of serum Lp-PLA2, Hcy, and color Doppler significantly improves the diagnostic accuracy, specificity, and susceptibility in the elderly with ACS, with little impact on their vascular endothelial function.

## 1. Introduction

Acute coronary syndrome (ACS) refers to a series of acute symptoms caused by changes in the position of plaques in the coronary arteries that affect the flow of blood in the arteries. Such symptoms can cause acute myocardial ischemia, myocardial infarction, angina, and thrombus [1–3]. The disease features a rapid onset and pronounced clinical symptoms, and delayed treatment may severely threaten the health and even the life of the patient. Elderly people are more susceptible to ACS, and the abnormality of blood pressure, blood lipids, blood sugar, and related indices indicate a high risk of ACS [4–6]. The diagnostic methods of ACS include imaging, blood index testing, and comprehensive detection. Color Doppler detection is a commonly used clinical detection method with high detection speed and can provide information on the internal conditions of blood vessels. Serum lipoprotein-associated phospholipase A2 is human plasma lipoprotein phospholipase A2 and contributes to the diagnosis of cardio-cerebral vascular embolism disease. Homocysteine (Hcy) is significantly correlated with the occurrence of cardiovascular events. It has been demonstrated that serum Hcy levels are directly proportional to the severity of coronary artery disease [7], and Hcy levels are also significantly higher in patients with ACS than in those without infarction. Studies have shown that hyperhomocysteinemia, triggered by abnormal Hcy metabolism, promotes the development of atherosclerosis and thrombosis, so Hcy demonstrates great potential as an independent risk factor for cardiovascular and cerebrovascular diseases [8–10]. To explore more reliable diagnostic methods for elderly patients with ACS, combined detection of serum levels of lipoprotein-associated phospholipase A2 (Lp-PLA2) and Hcy with color Doppler detection was performed in elderly patients with ACS in this study to evaluate their diagnostic value for ACS. Intensive treatment with statins is the mainstay of clinical treatment for ACS, but their hepatotoxicity restricts wide clinical application. In recent years, traditional Chinese medicine (TCM) has achieved great progress in the treatment of ACS, so patients with ACS herein were given a combination of self-prepared TCM decoction based on Western medical treatment to benefit Qi, activate blood circulation, and detoxify the blood.

## 2. Data and Methods

### 2.1. Materials

From February 2019 to October 2020, 100 elderly patients with suspected ACS enrolled in our hospital were recruited and assigned to either a control group (*n* = 50) or an experimental group (*n* = 50). In the control group, the patients in the control group were aged 66–79 years and in the experimental group were aged 65–80 years. There were no significant differences in terms of patient characteristics between the two groups (*P* > 0.05) (Table 1).

### 2.2. Inclusion or Exclusion Criteria

#### 2.2.1. Inclusion Criteria

Patients who were initially diagnosed as ACS; aged ≥ 60 years; with no history of drug allergy, no history of drug abuse, no bad habits; with no other organic diseases; who provided written informed consent were included [11]. The studies involving human participants were reviewed and approved by Cangzhou Central Hospital, No. CZ9817.

#### 2.2.2. Exclusion Criteria

Patients with a consciousness disorder that prevented treatment cooperation, who recently received surgical treatment, with unsuccessful emergency treatment were excluded.

### 2.3. Methods

Patients in the control group received color Doppler detection in a supine position, with a color Doppler ultrasound machine (Jiangsu Anmao Medical Technology Co. Ltd.; 20152221796; EPIQ7). The probe was placed at the arterial blood vessel and moved along the blood vessel with a frequency of 3–5 MHz. The blood flow velocity, the position of the atherosclerotic plaque, and the presence of embolisms in the blood vessel were observed. A similar color Doppler detection protocol was introduced to the patients in the experimental group.

Patients in the experimental group additionally received serum Lp-PLA2 and Hcy detection. Venous blood (5 ml) was collected from each patient, and then the levels of serum Lp-PLA2 and Hcy were determined by the enhanced immunoturbidimetric method. Diagnosis of the patients was made based on test results. The positive criteria were LP-PLA2 > 212.25 *μ*g/L, Hcy > 42.55 *μ*mol/L, and color Doppler monitoring, showing imaging features of ACS.

Treatment: the patients received 80 mg of simvastatin tablets (Merck Sharp & Dohme Pharmaceuticals Ltd., Lot No. 20140327) orally at bedtime daily for a fortnight. In addition, the patients also received 1 dose (400 mL) of Yiqi Huoxue Jiedu Decoction daily. The formula includes 15 *g* of Astragali Radix, 10 *g* of Ginseng, 15 *g* of Salviae Miltiorrhizae Radix et Rhizoma, 10 *g* of Chuanxiong Rhizoma, 5 *g* of leech, 10 *g* of Angelicae Sinensis Radix, 10 *g* of Forsythiae Fructus, 10 *g* of Corydalis Rhizoma, 10 *g* of Puerariae Lobatae Radix, 10 *g* of Lonicerae Japonicae Flos, and 10 *g* of licorice root. The above herbs were decocted with water to obtain 400 mL of filtrate, which was administered with a half dose administered in the morning and a half dose administered in the evening. The duration of treatment was a fortnight.

### 2.4. Indicators

The specificity, susceptibility, positive detection rate, negative detection rate, test accuracy, ROC-AUC, the expression levels of IL-2, IL-12, and IL-13, and the vascular endothelial function of the two selected groups were compared.

  Specificity = the number of diagnosed negative cases/the number of actual negative cases × 100%;
  Susceptibility = the number of diagnosed positive cases/the number of actual positive cases × 100%;
  Test accuracy = the number of detected cases/the number of confirmed cases × 100%.

Vascular endothelial function indices include prostaglandin I2 (PGI2), nitric oxide (NO), and tissue plasminogen activator (tPA). PGI2 relaxes blood vessels, NO has an anticoagulation effect, and tPA dissolves thrombus to a certain extent [12–14].

Patients with ACS were divided into three subgroups based on the Gensini score [15]: coronary artery disease stenosis <25% was counted as 1 point, that ≥25% and <50% as 2 points, that ≥50% and <75% as 4 points, that ≥75% and <90% as 8 points, that ≥90% and <99% as 16 points, and that ≥99% as 32 points. All the selected patients were separated into three groups: those with a score of 0–41 points were divided into the mild condition group, those with a score of 42–82 into the moderate condition group, and those with a score of 83–124 into the severe condition group. The Lp-PLA2 level and related laboratory indicators (fasting blood glucose, total cholesterol, triglyceride, high-density lipoprotein-cholesterol, low-density lipoprotein-cholesterol, apolipoprotein A-I, glutamic-pyruvic transaminase, lutamic-oxaloacetic transaminase, homocysteine, and amino-terminal pro-brain natriuretic peptide) were calculated.

### 2.5. Statistical Analysis

SPSS 20.0 was used for data analyses, and GraphPad Prism 7 (GraphPad Software, San Diego, USA) was used to plot the graphics. The measurement data are expressed as (mean ± SD) and analyzed using the *t*-test, and the count data are expressed (*n* (%)) and analyzed using the chi-square test. The multiple stepwise regression method was adopted in the multivariate analysis. *P* < 0.05 indicated that the difference was statistically significant.

## 3. Results

### 3.1. Positive and Negative Detection Results

Higher positive and negative detection rates were found in the experimental group than those in the control group (both *P* < 0.05) (Figure 1).

### 3.2. Specificity and Susceptibility

The experimental group had a more favorable outcome in terms of test susceptibility and specificity than the control group (both *P* < 0.05) (Figure 2).

### 3.3. Test Accuracy and AUC

The comparison results of the test accuracy and ROC-AUC between the two groups revealed higher levels of test accuracy and ROC-AUC in the experimental group (both *P* < 0.05) (Table 2 and Figure 3).

### 3.4. Expression Levels of IL-2, IL-12, and IL-13

There was no significant difference between the two groups of patients in terms of the levels of IL-2, IL-12, and IL-13 (all *P* > 0.05) (Figure 4).

### 3.5. Vascular Endothelial Function

There were no significant differences in the vascular endothelial function between the two groups of patients (*P* > 0.05) (Figure 5).

### 3.6. Lp-PLA2 Levels and Related Laboratory Indicators

There were no significant differences in the levels of fasting blood glucose, total cholesterol, triglyceride, HDL-C, low-density lipoprotein cholesterol ratio, apolipoprotein A1, alanine transaminase, aspartate transaminase (AST), Hcy, and N-terminal -pro hormone B-type natriuretic peptide (NT-proBNP) among the three subgroups (all *P* > 0.05). The severe condition group had the highest Lp-PLA2 level, followed by the moderate condition group, and then the mild condition group (*P* < 0.05) (Table 3).

### 3.7. Influencing Factors for the Coronary Gensini Score

With Fbg, lipoprotein (Lp(a)), ALT, AST, LDH, creatine kinase (CK), CK-MB, NT-proBNP, HCY, and Lp-PLA2 as independent variables, and coronary artery Gensini score as the dependent variable, multiple stepwise regression analysis was carried out. It was found that Lp-PLA2, aspartate transaminase, and NT-proBNP were all influencing factors for the Gensini score of ACS (all *P* < 0.05), and the equation was *Y* = −20.623 + 0.409 × Lp-PLA2 + 0.240 × AST + 0.006 × NT-proBNP (*P* < 0.05) (Table 4).

## 4. Discussion

ACS mostly occurs in elderly patients, and its risk factors include diabetes, hypertension, and hyperlipidemia. TACS develops when the plaque in the artery is dislodged or displaced after coronary atherosclerosis, which leads to blockage of the blood vessels and insufficient blood supply to the heart [15–17]. The onset of the disease is manifested by palpitations, angina pectoris, and myocardial ischemia, which requires timely treatment. Accurate diagnosis at admission to determine the type of disease and formulate targeted treatment is essential due to the potential overlap between the clinical presentation of cardiovascular disease and ACS [18–20]. At present, the most commonly used clinical diagnosis methods are color Doppler ultrasound diagnosis, CT, MRI diagnosis, and blood index testing, among which color Doppler ultrasound diagnosis is the simplest and fastest diagnosis method. Blood index testing facilitates the determination of related diseases by evaluation of the expression level of specific blood indices, which is associated with more accurate diagnostic results [21–23].

Results in the present study showed that the test specificity, susceptibility, positive detection, negative detection, test accuracy, and ROC-AUC in the experimental group were better than those in the control group (all *P* < 0.05), and there were no significant differences in the expression levels of IL-2, IL-12, IL-13, and the vascular endothelial function between the two groups (all *P* > 0.05). The results indicated that the color Doppler detection combined with serum Lp-PLA2 and Hcy diagnosis prominently increases the specificity, susceptibility, and accuracy of the test and thus significantly lowers the rate of misdiagnosis and missed diagnosis at admission. After the onset of ACS, the immediate removal of the plaques by surgical treatment is indispensable. Therefore, an accurate diagnosis of the patient's condition with the least delay possible is imperative to reduce the risk of surgery and treatment. In addition, endothelial function plays a crucial role in the human body, and vascular endothelial dysfunction is associated with various vascular diseases [7, 24]. Here, the results of the present research showed that the color Doppler detection cooperated with serum Lp-PLA2 and Hcy diagnosis had little impact on patients' endothelial function and levels of inflammatory factors, which indicated a high safety profile of the combined detection. Qian et al [25] revealed that the combined detection of serum Lp-PLA2 and Hcy levels could improve the accuracy of diagnosis and avoid missed diagnosis and misdiagnosis, which demonstrates a great application value for the early diagnosis of ACS, which was similar to the results in the present study. Moreover, there were no significant differences in the levels of Fbg, TC, TG, HDL-C, LDLC, ApoA1, ALT, AST, HCY, and NT-proBNP among the three subgroups (all *P* > 0.05). The severe condition group had the highest Lp-PLA2 level, followed by the moderate condition group, and the mild condition group (*P* < 0.05). Lp-PLA2, AST, and NT-proBNP were all influencing factors for the coronary Gensini score (*P* < 0.05). Carotid ultrasonography provides a comprehensive analysis of ACS in the elderly. Ultrasonography has high sensitivity and specificity through the enhancement of scattered echoes by the use of contrast agents, which enhances ultrasound diagnostic discrimination [1]. LP-PLA2 is a key indicator in the study of clinical vascular disease and an independent risk factor for cardiovascular disease mostly used to study inflammatory response mediators [2]. The pathological basis of ACS in the elderly is the rupture of coronary atherosclerotic plaque, followed by complete or incomplete occlusive thrombosis [3]. LP-PLA2 reflects the functional changes of the cardiovascular system, while carotid ultrasonography can visualize the lesion changes. Ultrasonography is preferred over conventional ultrasonography for the detection of specific lesions, with accurate detection of plaque properties and location, as well as new nuisance vessels within the plaque in elderly ACS [4]. It has been shown that ultrasonography could improve carotid plaque risk classification, and the combination with LP-PLA2 potentiates their effectiveness and further improve patient prognosis.

The combination of Yiqi Huoxue Jiedu Decoction with simvastatin intensive treatment reduces the TCM syndrome score in elderly ACS patients with Qi deficiency and blood stasis. In Yiqi Huoxue Jiedu Decoction, Astragali Radix tonifies Qi and protects the kidney [13], Ginseng tonifies blood, lung, and Qi, Salviae Miltiorrhizae Radix et Rhizoma activates blood circulation and resolves blood stasis, dilates blood vessels, inhibits platelet aggregation, and boosts anticoagulation, Chuanxiong Rhizoma moves Qi and relieves pain, Angelicae Sinensis Radix and Leech invigorate blood circulation [14], Forsythiae Fructus clears heat, detoxifies, disperses nodules and swelling, Puerariae Lobatae Radix relieves superficial fever and improves blood circulation [15], Lonicerae Japonicae Flos clears heat and detoxifies, and licorice root harmonizes all the herbs. The combination of all the herbs in this formula promotes the circulation of the ligaments, benefits the Qi, and removes toxins, thereby effectively decreasing the TCM syndrome score in elderly ACS patients [16, 17].

In conclusion, the combined detection of serum Lp-PLA2 and Hcy and color Doppler significantly improves the diagnostic accuracy, specificity, and susceptibility in the elderly with ACS, with little impact on their vascular endothelial function.

## Figures and Tables

**Figure 1:** Comparison of positive and negative detections between the two groups. The abscissa indicates the positive detection and the negative detection from left to right, and the ordinate indicates the number of cases. ^∗^indicates that 42 positive cases were detected in the experimental group, compared with 33 positive cases in the control group, *X*^2^ = 4.32, *P*=0.04, and the comparison result was statistically significant; ^∗∗^indicates that 8 cases were negative in the experimental group, compared with 1 case negative in the control group, *X*^2^ = 5.98, *P*=0.01, and the comparison result was statistically significant.

**Figure 2:** Comparison of the specificity and susceptibility between the two groups. The abscissa represents the specificity and susceptibility of the test from left to right, and the ordinate represents the specificity and susceptibility data. ^∗^indicates the significant difference between the test specificity of the experimental group ((91.51 ± 2.04) %) and that of the control group ((84.20 ± 1.59), %), *t* = 19.98, *P* < 0.001. ^∗∗^indicates the significant difference between the test susceptibility of the experimental group ((93.25 ± 2.11) %) and that of the control group ((81.07 ± 1.38) %), *t* = 34.16, *P* < 0.001.

**Figure 3:** Comparison of the test accuracy and AUC between the two groups.

**Figure 4:** Comparison of the expression levels of IL-2 and IL-12 between the two groups. (a) The abscissa represents IL-2, IL-12, and IL-13, respectively, and the ordinate represents the expression level (pg/ml). The insignificant difference between the IL-2 level of the experimental group ((26.65 ± 8.33) pg/ml) and that of the control group ((26.07 ± 8.28) pg/ml), *t* = 0.35, *P*=0.73. The insignificant difference between the IL-12 level of the experimental group ((33.58 ± 9.62) pg/ml) and that of the control group ((32.99 ± 9.41) pg/ml), *t* = 0.31, *P*=0.76. (b) The abscissa represents the experimental group and the control group, respectively, and the ordinate represents the expression level of IL-13 (pg/ml). The insignificant difference between the IL-13 level of the experimental group ((586.27 ± 99.80) pg/ml) and that of the control group ((589.34 ± 100.09) pg/ml), *t* = 0.15, *P*=0.88.

**Figure 5:** Comparison of PGI2, NO, and tPA level between the two groups. (a) The abscissa represents the experimental group and the control group, respectively, and the ordinate represents the expression level of PGI2 (*μ*mol/L). The insignificant difference between the PGI2 level of the experimental group ((66.70 ± 10.25) *μ*mol/L) and that of the control group ((66.98 ± 10.17) *μ*mol/L), *t* = 0.14, *P*=0.89. (b) The abscissa represents the experimental group and the control group, respectively, and the ordinate represents the expression level of NO (pg/L). The insignificant difference between the NO level of the experimental group ((25.88 ± 5.91) pg/L) and that of the control group ((25.03 ± 5.87) pg/L), *t* = 0.72, *P*=0.47. (c) The abscissa represents tPA and the ordinate indicates the expression level (ng/L). The insignificant difference between the tPA level of the experimental group ((17.83 ± 2.21) ng/L) and that of the control group ((17.91 ± 2.30) ng/L), *t* = 0.18, *P*=0.47.

**Table 1:** General data comparison statistics.

Group	Experimental group	Control group	*X* ^2^/*t*	*P* value
Gender (male/female)	23/27	26/24	0.36	0.55
Age (year-old)	73.34 ± 5.52	73.77 ± 5.39	0.39	0.69
Height (cm)	166.52 ± 10.91	166.80 ± 10.26	0.13	0.90
Weight (kg)	69.29 ± 5.88	69.34 ± 5.64	0.04	0.97
Medical time (h)	1.68 ± 0.69	1.72 ± 0.73	0.28	0.78
Smoking history (year)	6.61 ± 1.33	6.57 ± 1.38	0.15	0.88
Drinking history (year)	9.96 ± 1.38	9.88 ± 1.65	0.26	0.79
Hypertension (number of cases)	13	15	0.20	0.66
Diabetes (number of cases)	8	7	0.08	0.78
Hyperlipidemia (number of cases)	4	6	0.44	0.51

**Table 2:** Comparison of the test accuracy and AUC between the two groups ($\bar{\text{x}}$ ± *s*).

Group	Test accuracy (%)	AUC
Experimental group	100%	0.85 ± 0.10
Control group	79%	0.66 ± 0.09
*X* ^2^/*t*	23.46	9.99
*P* value	<0.001	<0.001

**Table 3:** Lp-PLA2 levels and other laboratory indicators related to the Gensini score.

Index	Mild condition group (*n* = 16)	Moderate condition group (*n* = 17)	Severe condition group (*n* = 16)	*F*	*P* value
Fbg (mmol/L)	5.71 ± 2.91	5.75 ± 2.03	5.25 ± 1.87	0.036	0.964
TC (mmol/L)	4.01 ± 1.16	3.97 ± 0.88	4.16 ± 0.94	0.18	0.835
TG (mmol/L)	1.73 ± 1.11	1.59 ± 0.76	1.60 ± 0.63	0.259	0.772
HDL-C (mmol/L)	1.13 ± 0.27	1.15 ± 0.27	1.14 ± 0.23	0.071	0.932
LDLC (mmol/L)	2.18 ± 0.61	2.19 ± 0.64	2.39 ± 0.65	0.553	0.577
ApoA1 (g/L)	1.09 ± 0.19	1.10 ± 0.11	1.05 ± 0.15	0.608	0.546
ALT (U/L)	32.36 ± 21.78	30.15 ± 21.12	43.71 ± 27.90	1.92	0.152
AST (U/L)	38.23 ± 29.53	47.77 ± 33.89	60.64 ± 31.09	2.877	0.061
NT-proBNP (ng/L)	331.59 ± 58.40	467.56 ± 76.11	958.36 ± 155.51	3.055	0.052
HCY (*μ*mol/L)	15.05 ± 7.57	16.95 ± 11.64	22.48 ± 18.35	2.297	0.106
Lp-PLA2 (*μ*g/L)	121.07 ± 30.72	139.82 ± 32.35a	172.13 ± 34.72ab	14.024	<0.001

a: compared to the mild condition group,*P* < 0.05; b: compared to the moderate condition group, *P* < 0.05.

**Table 4:** Influencing factors for coronary Gensini scores.

Indicators	Partial regression coefficient	Standard error	Beta	*t*-value	*P* value
Lp-PLA2 (*μ*g/L)	0.424	0.027	0.613	9.457	<0.001
AST (U/L)	0.211	0.075	0.352	3.11	0.002
NT-proBNP (*μ*mol/L)	0.015	0.001	0.245	2.123	0.001

## Data Availability

All the data generated or analyzed during this study are included in this published article.
